The article "Application Value of Real-Time Ultrasonic Elastograph with Serum Human Epididymis Protein 4, Interleukin-33, and Carbohydrate Antigen 153 in Diagnosis of Early Cervical Cancer" was retracted in 2023. Reason: concerns about the peer review.

# Application Value of Real-Time Ultrasonic Elastograph with Serum Human Epididymis Protein 4, Interleukin-33, and Carbohydrate Antigen 153 in Diagnosis of Early Cervical Cancer

**DOI:** 10.1155/2022/4880874

**Published:** 2022-04-12

**Authors:** Maoping Guo, Lingling Liang, Litao Wu, Daolin Xie, Jian Li

**Affiliations:** ^1^Department of Ultrasound, Affiliated Heji Hospital of Shanxi Changzhi Medical College, Changzhi City 046000, Shanxi Province, China; ^2^Department of Gynecology, Affiliated Heji Hospital of Shanxi Changzhi Medical College, Changzhi City 046000, Shanxi Province, China

## Abstract

**Objective:**

To explore the application value of real-time ultrasonic elastograph (USE) with serum human epididymis protein 4 HE4, interleukin-33 (IL-33), and carbohydrate antigen 153 (CA153) in the diagnosis of early cervical cancer.

**Methods:**

A total of 120 cervical cancer patients treated in our hospital (06, 2019–06, 2021) and meeting the study criteria were screened and divided into the benign group (BG, *n* = 70) and malignant group (MG, *n* = 50) according to their final diagnostic results, and healthy females who received physical examination in our hospital in the same period were selected as the control group (CG, *n* = 60). Patients in the three groups received real-time USE and detection of serum HE4, IL-33, and CA153 so as to analyze the diagnostic value of single examination and combined examination in diagnosing early cervical cancer.

**Results:**

The patients' real-time USE score, *E*_max_, *E*_mean_, and elastic fibers were significantly higher in the MG than those in the BG (*P* < 0.05), and the patients' real-time USE *E*_min_, stroma ratio and collagen fibers were significantly lower in the MG than those in the BG (*P* < 0.05); the HE4, IL-33, and CA153 levels were obviously higher in the MG than those in the BG (*P* < 0.05) and were significantly higher in the BG than those in the CG (*P* < 0.05); the positive detection rate of combining real-time USE with serum HE4, IL-33, and CA153 was higher than that of single examination, and the diagnostic accuracy rate, sensitivity, specificity, positive predictive value, and negative predictive value of the combined examination were significantly higher than those of single examination (*P* < 0.05); according to the diagnostic efficacy of single examination and combined examination in diagnosing early cervical cancer by ROC curve, it was combined diagnosis > real-time USE > HE4 > CA153 > IL-33.

**Conclusion:**

Combined examination of real-time USE and serum HE4, IL-33, and CA153 has higher diagnostic value in diagnosing early cervical cancer, which can obviously improve the diagnostic accuracy rate of cervical cancer.

## 1. Introduction

Cervical cancer is one of the common malignant tumors of the female reproductive system in China, which causes serious harm to the physical health and life of Chinese women. According to clinical statistics, squamous epithelial carcinoma accounts for approximately 90% of cervical cancer, and adjacent tissue invasion and metastasis are relatively common [1–4]. At present, surgery is still the main means of treating cervical cancer, and neoadjuvant chemotherapy is also widely recognized, but the early symptoms of cervical cancer are not typical and can be easily ignored, so corresponding clinical symptoms often present when patients are at the middle to late stage, causing great distress to the affected women. Therefore, a retrospective study on the early diagnosis of cervical cancer was conducted herein, aiming to promote the diagnosis efficiency of early cervical cancer and guide prognosis to improve patient survival. Currently, the main modalities for clinical screening and diagnosis of cervical cancer include colposcopic gynecological examination, liquid-based thin-cytology test (TCT), HPV testing, and biopsy [5, 6]. TCT and colposcopy are important methods for the diagnosis of cervical intraepithelial neoplasia and early invasive cervical cancer, but with multiple affecting factors such as cervical morphology, lesion type, and subjectivity of the operator, their false negative rate for early detection is high. In addition, conventional ultrasonography can observe the size, morphology, space occupying range, blood flow, and relationship with surrounding tissues, but it has some limitations in the qualitative diagnosis of cervical lesions. In recent years, transvaginal ultrasound elastograph (USE), as an emerging ultrasound diagnosis technique, is able to provide information on the stiffness of tissues and improve the diagnostic accuracy rate of cervical cancer, but some studies have pointed out that erroneous diagnosis and missed diagnosis may occur in some patients when diagnosing cervical cancer by USE, for example, patients with tumor hemorrhage and necrosis, formation of calcification focus, changes in tissue hardenability, or too small focus [7, 8]. Based on this, researchers found that the detection of human epididymis protein 4 (HE4), interleukin-33 (IL-33), and carbohydrate antigen 153 (CA153) has a certain value in diagnosis cervical cancer and can assist in the definite diagnosis and follow-up, which provides a new research idea and direction for the early diagnosis of cervical cancer. Combining such detection with real-time USE is expected to improve the diagnostic efficacy of early cervical cancer. Therefore, the application value of combining real-time USE with serum HE4, IL-33, and CA153 in diagnosing early cervical cancer was explored herein, in the hope of providing reference for establishing clinical treatment scheme and patient condition evaluation.

## 2. Materials of Patients

### 2.1. Cases Screening

The inclusion criteria and exclusion criteria were proposed according to the study objective. Inclusion criteria are as follows: (1) The patients met the clinical diagnosis criteria for cervical cancer [9] and were diagnosed after imaging examination, laboratory examination, and according to their clinical manifestations; (2) the patients received pathological examination after surgery, which was regarded as the gold standard; (3) the patients had complete clinical data and were diagnosed in our hospital for the first time; and (4) the patients and their family members understood the study and signed the informed consent. Exclusion criteria for patients are as follows: (1) complicated with lesions in the brain, heart, kidney, liver, and other organs and tissues; (2) complicated with other malignant tumors; (3) pregnant or lactating women; (4) presence of seeing-hearing disorder or cognitive disorder; (5) low compliance; and (6) with history of chemoradiotherapy or surgical treatment. On this basis, 120 cervical cancer patients treated in our hospital (06, 2019–06, 2021) and meeting the study criteria were screened as the study objects.

### 2.2. Grouping

The screened 120 cervical cancer patients were divided into the benign group (BG, *n* = 70) and malignant group (MG, *n* = 50) according to the final diagnosis results, and healthy women who received physical examination in our hospital in the same period were selected as the control group (CG, *n* = 60); and the study met the World Medical Association Declaration of Helsinki (2013) [10].

## 3. Methods

### 3.1. Real-Time USE

The color Doppler ultrasonic diagnostic apparatus (model: Philips EPIQ7) that is equipped with USE technique was used, with the probe frequency of 4–15 MHz. Before surgery, the patients received real-time USE examination and serum specimen detection. Real-time USE examination: patients were lying on the back to expose the cervical part for routine ultrasonic examination first, the probe was vertical to the body surface and slowly moved, after finding the location of lesion, the patients were asked to hold their breath for 3 s to stabilize the image, and the ultrasound probe axis was swept along the direction vertical to the cervix to the surrounding so as to check the tissues of the whole cervix [11]. After the image was stabilized, it was switched to the elastograph imaging mode, the part 3–4 times of lesion site was regarded as the key observation area to carefully explore the lesion zone and its margins for echogenicity and decomposition and check if there was lymphatic metastasis under both arms, thus implementing probe pressurization and decompression to obtain stable elastic images, which were evaluated by the 1–5 point method.

### 3.2. Detection of Serum Markers

Three to five ml of fasting blood specimens were taken from patients in the early morning to detect their HE4, IL-33, and CA153 levels by using the automatic electrochemiluminescence immune analyzer (manufactured: Roche Company) in strict accordance with the specification.

### 3.3. Observation Indicators

Scoring criteria for real-time USE [12]: 1 point indicated that the lesion or tissue was shown as green or blue in a whole; 2 points indicated that center of lesion was shown as green and its peripheral tissue was blue; 3 points indicated that mixed green and blue in the lesion, and the proportion of the two colors differed little; 4 points indicated that the lesion was shown as red or with a little green as a whole; and 5 points indicated that the lesion was shown as red in a whole, and its peripheral tissue was shown as blue, with or without green.

Determination criteria for serum markers: HE4 ≥ 140 pmol/ml, IL-33 ≥ 230 *μ*g/L, and CAl53 ≥ 25 U/ml indicated cervical cancer positive; in combined diagnosis, cervical cancer positive could be diagnosed in case of single indicator positive [13].

### 3.4. Statistical Processing

In this study, the between-group differences of data were calculated by SPSS22.0, the picture drawing software was GraphPad Prism 7 (GraphPad Software, San Diego, USA), the items included were enumeration data and measurement data, which were expressed by *n* (%) and ($\bar{x}\pm s$) and examined by *X*^2^ test and *t*-test, respectively, and differences were considered statistically significant at *P* < 0.05.

## 4. Results

### 4.1. General Data

No statistical differences in patients' age, BMI, lesion diameter, FIGO staging, educational degree, history of gynecological diseases, and family medical history among the three groups were observed (*P* > 0.05) (see Table 1).

### 4.2. Diagnostic Results of Real-Time USE

The patients' real-time USE score, *E*_max_, *E*_mean_, and elastic fibers were significantly higher in the MG than those in the BG (*P* < 0.05), and the patients' real-time USE *E*_min_, stroma ratio, and collagen fibers were significantly lower in the MG than those in the BG (*P* < 0.05) (see Tables 2 and 3).

### 4.3. Serum HE4, IL-33, and CA153 Levels

According to the statistics in Table 4, the HE4, IL-33, and CA153 levels were obviously higher in the MG than those in the BG (*P* < 0.05) and were significantly higher in BG than in CG (*P* < 0.05).

### 4.4. Diagnostic Efficacy of Single Examination and Combined Examination

According to Tables 5 and 6, the positive detection rate of combining real-time USE with serum HE4, IL-33, and CA153 was higher than that of single examination, and the diagnostic accuracy rate, sensitivity, specificity, positive predictive value (PPV), and negative predictive value (NPV) of the combined examination were significantly higher than those of single examination (*P* < 0.05); according to the diagnostic efficacy of single examination and combined examination in diagnosing early cervical cancer by ROC curve (see Figure 1 and Table 7), it was combined diagnosis > real-time USE > HE4 > CA153 > IL-33.

## 5. Discussion

With the progress of China's mass examination on cancer, the diagnostic rate of early cervical cancer in China has gradually increased, which is associated with enhanced health education, HPV vaccination, and cervical cancer screening. However, the cervical cancer-related data released by WHO in 2018 showed that there is an obvious decreasing trend in the incidence and case fatality of cervical cancer worldwide in the past 40 years, and a decreasing average age of onset and a clear tendency that there are more and more young cervical cancer patients [14, 15]. Currently, ultrasonography is the main diagnosis modality for cervical cancer, and USE refers to the modality based on routine ultrasound with additional data information on tissue stiffness, when clinical diagnosis is made, real-time USE can show tissue stiffness and the deformation degree of tissue after being stressed, and transform the amplitude of echo signal change before and after tissue compression into real-time color images to show elastography of tissues. This examination method to some extent compensates for the inadequacy of conventional ultrasound, improves the sensitivity and specificity of clinical diagnosis of cervical cancer, with the advantages of noninvasion and low cost [16–19]. In this study, the real-time USE provided the elastic index and relevant parameters of cervical cancer lesion, and the lesion stiffness was evaluated by the 5-point scoring method. The study results showed that the patients' real-time USE score, *E*_max_, *E*_mean_, and elastic fibers were significantly higher in the MG than those in the BG (*P* < 0.05), and the patients' real-time USE *E*_min_, stroma ratio and collagen fibers were significantly lower in the MG than those in the BG (*P* < 0.05), which were consistent with the report by Sanchez et al. [20], confirming that data such as the real-time USE parameters and stroma were obviously different in benign and malignant cervical cancer lesions. From the pathogenesis point of view, stiffness is one of the important biomechanical characteristics of tissue. Malignant lesion tissue adhesion with nearby structures leads to reduced mobility, and thus the tissue is stiffer than the surrounding normal tissue and has complex internal component, while benign lesion tissue is softer and has single internal component, so the maximum value of intralesional stiffness is able to reflect the actual stiffness of the lesion. However, there are also many patients who have some heterogeneous components in their lesions, and this diagnostic method is susceptible to subjective factors from physicians and lacks quantifiable criteria in disease diagnosis, which, combined with the very complex internal stromal components in cervical cancer lesions with soft or hard texture, such as liquefactive necrosis area and malignant tissue, results in certain false negatives or false positives when diagnosing cervical cancer.

Moreover, HE4, IL-33, and CA153 indicators were included in the study to further improve the accuracy rate of diagnosing early cervical cancer. Among them, HE4 is an epididymis specific-related protein and a novel tumor marker, which inhibits serine protease and is directly involved in the protection against microorganisms in the body and is also able to have an effect on cell growth and differentiation. Meanwhile, HE4 can stimulate the production of vascular endothelial growth factor as well as matrix metalloproteinases in the body, accelerating lesion tissue vascularization as well as extracellular matrix degradation and inducing tumor growth. Zhang et al. [14] reported that endometrium, fallopian tube, and cervix were the main sources of HE4 in healthy tissues, but the level of HE4 in healthy tissues was low and its expression was significantly higher in malignant tissues. CA153 is an important tumor marker for cervical cancer detection in the clinic and is mainly used for monitoring of cervical cancer recurrence and metastasis. IL-33 is normally released upon epithelial cell injury or necrosis, and IL-33 in tumor cells induces epithelial to mesenchymal transition by activating the ST2 receptor, which in turn promotes tumorigenesis; IL-33 can further activate the nuclear factor-*κ*B signaling pathway upon activation of ST2 receptor, which promotes matrix metalloproteinase-3 expression and then drives tumorigenesis and metastasis; in addition, IL-33 also inhibits T cell function and promotes tumor tissue angiogenesis and local infiltration [21–24]. In this study, the HE4, IL-33, and CA153 levels in patients were obviously higher in the MG than those in the BG (*P* < 0.05) and were significantly higher in the BG than those in the CG (*P* < 0.05), implying that serum HE4, IL-33, and CA153 markers have certain value in early screening of cervical cancer and can reflect patients' condition. Besides, the positive detection rate of combining real-time USE with serum HE4, IL-33, and CA153 was higher than that of single examination, and the diagnostic accuracy rate, sensitivity, specificity, PPV, and NPV of the combined examination were significantly higher than those of single examination (*P* < 0.05); according to the diagnostic efficacy of single examination and combined examination in diagnosing early cervical cancer by ROC curve, it was combined diagnosis > real-time USE > HE4 > CA153 > IL-33, implying that combined diagnosis has higher application value in early diagnosis of cervical cancer, can make up for the disadvantages of single method, and provides strong reference for diagnosing cervical cancer. Limited by the time cost and economic cost, the sample size of the study was small, so large sample data are required for future verification and analysis.

In conclusion, combining real-time USE with serum HE4, IL-33, and CA153 has higher diagnostic value in early cervical cancer and can obviously improve the diagnostic accuracy rate of cervical cancer.

## Figures and Tables

**Figure 1:** ROC curves.

**Table 1:** Comparison of patients' general data among the three groups.

Observation indicator	MG (*n* = 50)	BG (*n* = 70)	CG (*n* = 60)	*P* value

Age (years)	44.56 ± 3.55	45.82 ± 4.13	45.69 ± 3.35	>0.05
BMI (kg/m^2^)	23.42 ± 2.18	23.36 ± 3.01	23.55 ± 2.40	>0.05
Lesion diameter (mm)	25.53 ± 3.35	25.76 ± 3.28	—	>0.05
FIGO staging				
I	35 (70)	47 (67.14)	—	>0.05
II	15 (30)	23 (32.86)	—	
Educational degree				
Below senior high school	14 (28)	20 (28.57)	17 (28.33)	>0.05
Senior high school	21 (42)	28 (40)	24 (40)	>0.05
Above senior high school	15 (30)	22 (31.43)	19 (31.67)	>0.05
History of gynecological diseases				
Yes	12 (24)	22 (31.43)	17 (28.33)	>0.05
No	38 (76)	48 (68.57)	43 (71.67)	
Family medical history				
Yes	3 (6)	9 (12.86)	7 (11.67)	>0.05
No	47 (94)	61 (87.14)	53 (88.33)	

FIGO staging is the staging criteria of International Federation of Gynecology and Obstetrics for gynecologic tumors; which classifies tumors into 4 stages, of which stage I refers to tumors confined to the vulva or perineum, the maximum diameter of lesions ≤2 cm, and no metastasis to lymph nodes; stage II refers to the tumors confined to the vulva or perineum, the maximum diameter of lesions >2 cm, and no metastasis to lymph nodes. So, stage I and II patients met the setting of this study for early cervical cancer.

**Table 2:** Real-time USE scores.

Score	MG (*n* = 50)	BG (*n* = 70)	*t*/*X*^2^	*P* value

0 point	0 (0)	9 (12.86)	6.950	0.008
1 point	0 (0)	21 (30)	18.182	<0.001
2 points	0 (0)	35 (50)	35.294	<0.001
3 points	8 (16)	5 (7.14)	2.369	0.124
4 points	28 (56)	0 (0)	51.130	<0.001
5 points	14 (28)	0 (0)	22.189	<0.001
Mean score	4.12 ± 0.65	1.51 ± 0.81	18.851	<0.001

**Table 3:** Real-time USE parameters and stroma component.

Parameter and stroma	MG (*n* = 50)	BG (*n* = 70)	*t*	*P* value

*E*_max_	133.85 ± 32.16	50.95 ± 9.41	20.408	<0.001
*E*_min_	0.13 ± 0.02	3.11 ± 0.75	28.044	<0.001
*E*_mean_	28.75 ± 4.26	15.03 ± 2.01	23.551	<0.001
Stroma ratio (%)	44.36 ± 10.25	64.53 ± 10.11	10.713	<0.001
Collagen fibers (%)	56.15 ± 10.55	62.13 ± 10.29	3.106	0.002
Elastic fibers (%)	23.05 ± 6.87	12.83 ± 4.64	9.729	<0.001

**Table 4:** Patients' HE4, IL-33, and CA153 levels of the three groups.

Group	*n*	HE4 (pmol/ml)	IL-33 (*μ*g/L)	CA153 (U/ml)

MG	50	149.71 ± 12.08^*∗*#^	280.94 ± 15.17^*∗*#^	44.15 ± 9.20^*∗*#^
BG	70	128.15 ± 9.33^*∗*^	217.46 ± 12.13^*∗*^	20.03 ± 5.24^*∗*^
CG	60	75.24 ± 8.25	153.60 ± 10.17	15.88 ± 2.83

^*∗*^Statistically significant difference compared with CG (*P* < 0.05); ^#^Statistically significant difference compared with BG (*P* < 0.05).

**Table 5:** Comparison with pathologic findings.

Pathologic findings	*N*	Combined diagnosis		USE		HE4		CA153		IL-33	
		+	−	+	−	+	−	+	−	+	−

+	50	47	3	46	4	45	5	42	8	38	12
−	70	4	66	5	65	6	64	10	60	14	56

**Table 6:** Analysis on diagnostic value of single examination and combined diagnosis on cervical cancer.

Examination indicator	Accuracy rate	Sensitivity	Specificity	PPV	NPV

Combined examination	94.17	94.00	94.29	92.16	95.65
Real-time USE	92.50	92.00	92.86	90.20	94.20
HE4	90.83	90.00	91.43	88.24	92.75
CA153	85.00	84.00	85.71	80.77	88.24
IL-33	78.33	76.00	80.00	73.08	82.35

**Table 7:** Area under curve.

Test results variables	Area	SE^a^	Asymp. Sig.^b^	Asymp. 95% CI

Combined examination	0.941	0.025	0.000	0.892–0.991
Real-time USE	0.924	0.029	0.000	0.868–0.980
HE4	0.907	0.031	0.000	0.846–0.969
CA153	0.849	0.039	0.000	0.773–0.924
IL-33	0.780	0.045	0.000	0.692–0.868

^a^Under nonparametric hypothesis; ^b^Null hypothesis: solid area = 0.5; Sig: significance, indicating the “significance level.”

## Data Availability

The data to support the findings of this study are available on reasonable request from the corresponding author.
